The article "Application of Bayesian Decision Tree in Hematology Research: Differential Diagnosis of β-Thalassemia Trait from Iron Deficiency Anemia" was published in 2021. Journal: Comput Math Methods Med.

# Application of Bayesian Decision Tree in Hematology Research: Differential Diagnosis of *β*-Thalassemia Trait from Iron Deficiency Anemia

**DOI:** 10.1155/2021/6401105

**Published:** 2021-11-09

**Authors:** Mina Jahangiri, Fakher Rahim, Najmaldin Saki, Amal Saki Malehi

**Affiliations:** ^1^Ph.D. Student, Department of Biostatistics, Faculty of Medical Sciences, Tarbiat Modares University, Tehran, Iran; ^2^Thalassemia & Hemoglobinopathy Research Center, Research Institute of Health, Ahvaz Jundishapur University of Medical Sciences, Ahvaz, Iran; ^3^Department of Biostatistics and Epidemiology, Faculty of Public Health, Ahvaz Jundishapur University of Medical Sciences, Ahvaz, Iran

## Abstract

**Objective:**

Several discriminating techniques have been proposed to discriminate between *β*-thalassemia trait (*β*TT) and iron deficiency anemia (IDA). These discrimination techniques are essential clinically, but they are challenging and typically difficult. This study is the first application of the Bayesian tree-based method for differential diagnosis of *β*TT from IDA.

**Method:**

This cross-sectional study included 907 patients with ages over 18 years old and a mean (±SD) age of 25 ± 16.1 with either *β*TT or IDA. Hematological parameters were measured using a Sysmex KX-21 automated hematology analyzer. Bayesian Logit Treed (BLTREED) and Classification and Regression Trees (CART) were implemented to discriminate *β*TT from IDA based on the hematological parameters.

**Results:**

This study proposes an automatic detection model of beta-thalassemia carriers based on a Bayesian tree-based method. The BLTREED model and CART showed that mean corpuscular volume (MCV) was the main predictor in diagnostic discrimination. According to the test dataset, CART indicated higher sensitivity and negative predictive value than BLTREED for differential diagnosis of *β*TT from IDA. However, the CART algorithm had a high false-positive rate. Overall, the BLTREED model showed better performance concerning the area under the curve (AUC).

**Conclusions:**

The BLTREED model showed excellent diagnostic accuracy for differentiating *β*TT from IDA. In addition, understanding tree-based methods are easy and do not need statistical experience. Thus, it can help physicians in making the right clinical decision. So, the proposed model could support medical decisions in the differential diagnosis of *β*TT from IDA to avoid much more expensive, time-consuming laboratory tests, especially in countries with limited recourses or poor health services.

## 1. Introduction

Iron deficiency anemia (IDA) and *β*-thalassemia trait (*β*TT) are the two most common hypochromic microcytic anemia. *β*TT is more prevalent in the Mediterranean region, in specific geographical areas, including the Caspian Sea and Persian Gulf regions; the 10% prevalence was reported [1]. The differential between *β*TT from IDA is crucial for preventing iron overload and related complications caused by misdiagnosis and inaccurate treatment [2].

Differentiation of *β*-thalassemia trait from iron deficiency anemia is also essential for premarital counseling in developed countries; for patients with microcytic anemia, complete blood count (CBC), in conjunction with hemoglobin variant analysis by high-performance liquid chromatography (HPLC), is interpreted to differentiate iron deficiency from thalassemia traits. Then, iron studies and molecular testing are also performed. Hemoglobin electrophoresis, serum iron, and ferritin levels are considered to make a definitive differential diagnosis between *β*TT and IDA [3–5].

However, in low-resource settings where HPLC and molecular testing are not available, different studies proposed discrimination indices to distinct between *β*TT and IDA. These indices have been defined to quickly discriminate between IDA and *β*TT and avoid more time-consuming and expensive methods. Mentzer [3], Shine and Lal [4], England and Fraser [5], RBC [6], Srivastava and Bevington [7], Ricerca et al. [8], Green and King [9], Bessman and Feinstein (RDW) [10], Gupta et al. [11], Jayabose et al. (RDWI) [12], Telmissani-MCHD [13], Telmissani-MDHL [13], Huber-Herklotz [14], Kerman I [15], Kerman II [15], Sirdah et al. [16], Ehsani et al. [17], Keikhaei [18], Nishad et al. [19], Wongprachum et al. [20], Dharmani et al. [21], Pornprasert et al. [22], Sirachainan et al. [23], Bordbar et al. [24], Matos et al. [25], Janel (11T) [26], CRUISE Index [27], and Index26 [27] are all hematological discrimination indices used for discriminating between the IDA and the *β*TT. However, these indices were obtained empirically and have an inconsistent performance for differential diagnosis of *β*TT and IDA in the same patient [28]. On the other hand, sometimes, the same indices showed different discrimination power in varied age groups [29, 30].

Recently, the accessibility of powerful statistical software has provided data mining techniques for health-related data. Many studies have proposed advanced statistical methods and data mining techniques such as decision tree methods [31] for differential diagnostic between *β*TT and IDA to avoid much more expensive, time-consuming, and complicated laboratory procedures and nonsatisfactory hematological indices in discriminating between *β*TT and IDA [32–38]. [32, 35–39]. Urrechaga, Aguirre, and Izquierdo [39] used multivariable discriminant analysis for differential diagnosis of microcytic anemia. Wongseree et al. [37] implemented neural network and genetic programming for thalassemia classification. Dogan and Turkoglu [35] proposed a decision tree for detecting iron deficiency anemia from hematology parameters.

Jahangiri et al. [32] used classic decision-tree-based methods for constructing a differential diagnosis scheme and investigating the performance of several tree-based methods for the differential diagnosis of *β*TT from IDA. Decision trees have advantages over traditional statistical methods like discriminant analysis and generalized linear models (GLMs). The main advantage of tree-based methods is a tree structure that makes it easy to interpret the clinical data and be accepted by medical researchers and clinicians. CART is one of the best-known classic tree algorithms. However, this algorithm suffers from some problems such as greediness, instability, and bias in split rule selection. Bayesian tree approaches were proposed to solve the greediness of the CART algorithm. The greedy search algorithm has disadvantages such as limit the exploration of tree space, the dependence of future splits to previous splits, generate optimistic error rates, and the inability of the search to find a global optimum [40]. Also, the Bayesian approaches can quantify uncertainty and explore the tree space more than classic tree approaches. Bayesian approaches combine prior information with observations, unlike classic tree methods (these methods use only observations for data analysis). The Bayesian approaches define prior distributions on the components of classic tree methods and then use stochastic search algorithms through Markov Chain Monte Carlo (MCMC) algorithms for exploring tree space [41–47]. So, in the last two decades, many studies have developed Bayesian Treed Generalized Linear Models. These models fit a parametric model such as GLMs instead of using constant models in each tree node. So, these treed algorithms create smaller trees than tree models and improve the tree's interpretation [43].

This paper aims to compare the Bayesian Treed Generalized Linear Models and CART for the differential diagnosis of *β*TT from IDA based on simple laboratory test results. The outcome variable of the present study is qualitative, so we must use the Bayesian Logit Treed (BLTREED) algorithm for discrimination between these two disorders. This Bayesian treed model fits the logistic regression model in each tree node for data prediction and uses the Metropolis-Hastings algorithm for exploring tree space.

## 2. Material and Methods

### 2.1. Criteria for Selecting Patient Groups

In this study, a total of 907 patients aged over 18 years old diagnosed with IDA (*n* = 370) or *β*TT (*n* = 537) were selected. The mean (±SD) age of the patients was 25 ± 16.1 years. Most of the patients (*n* = 592 (65%)) were women, and 315 (35%) were men.

CBC analysis of EDTA-K2 anticoagulated blood samples was performed using the Sysmex KX-21 automated hematology analyzer (Japan) to measure differential parameters. Hematological parameters like hemoglobin (Hb), mean corpuscular volume (MCV), mean corpuscular hemoglobin (MCH), Red Blood Cell Distribution Width (RDW), Mean Corpuscular Hemoglobin Concentration (MCHC), and Red Blood Cell count (RBC) were measured for all patients.

### 2.2. Inclusion Criteria

In the IDA group, patients had hemoglobin (Hb) levels less than 12 and 13 g/dl for women and men, respectively. Mean corpuscular hemoglobin (MCH) and mean corpuscular volume (MCV) were below 80 fl and 27 pg for both sexes, respectively, and for men, ferritin of <28 ng/ml was considered as IDA. In the *β*TT group, patients had an MCV value below 80 fl. Patients with HbA2 levels of >3.5% were considered as *β*TT carriers.

### 2.3. Exclusion Criteria

In the IDA group, the patients who had mutations associated with *α*TT (3.7, 4.2, 20.5, MED, SEA, THAI, FIL, and Hph) were excluded. For the *β*TT group, patients with *α*TT confirmed by mutations in the molecular analysis were excluded. All patients with malignancies or inflammatory/infectious diseases were also excluded.

### 2.4. Ethical Consideration

This study was approved and supported by the Ethical committee affiliated with the Ahvaz Jundishapur University of Medical Sciences (AJUMS), Ahvaz, Iran. Written informed consent was filled before the enrollment.

### 2.5. Machine Learning Analysis

Tree-based machine-learning methods are valuable tools in data mining techniques. These methods empower predictive models and could provide a solution for constructing the diagnostic test with high accuracy [48, 49]. Tree-based models do not need any assumptions about the functional form of the data.

One of the advantages of these methods is the graphical presentation of results that make them easy to interpret and no need for statistical experience for the understanding result of models [50–53]. Tree-based models also were constructed based on Bayesian algorithms. Chipman et al. proposed the Bayesian approach of the CART model (BCART) with defining a prior distribution. Chipman et al. also developed the Bayesian Logit Treed (BLTREED) model as an extension of BCART. The BLTREED model fits a logistic regression model for data prediction in the terminal nodes [43, 54].

#### 2.5.1. Bayesian Logit Treed (BLTREED) Model

The Bayesian approach (BCART) was implemented by using a prior distribution on the two components (Θ, *T*) of the CART model; *T* is a binary tree with *𝒦* terminal nodes or tree with size *𝒦*, and Θ = (*θ*_1_, *θ*_2_, ⋯, *θ*_*𝒦*_) is the parameter set in the terminal nodes (*θ*_*i*_ = *p*_*ij*_, *i* = 1, ⋯, *𝒦*, *j* = 1, ⋯, *N*: the number of distinct classes of the response variable and *p*_*ij*_ shows the probability of the *j*th class of response variable in *i*th terminal node). The joint posterior distribution of parameters and tree structure was as the following equation:

(1) $$\begin{array}{c} p\left(\Theta ,T\right)=p\left(\Theta \left|T\right.\right)p\left(T\right), \end{array}$$

where *p*(*T*) and *p*(Θ | *T*) show the prior distributions for tree and parameters in terminal nodes, respectively.

Usually, the Bayesian approach defines prior distributions as unknown; so, tree structure and parameters in terminal nodes were considered unknown [42]. BCART was extended by fitting a parametric model such as a logistic regression model for data prediction and describing the conditional distribution of *Y*|*X* in each terminal node [43, 54]. In the BLTREED model, the conditional distribution of *Y*|*X*, unlike the BCART model, depends on *X* (*Y* | *X* ~ *f*(*Y* | *X*, *θ*_*i*_)) and also by fitting sophisticated model at terminal nodes (by fitting logistic regression model for data prediction in each terminal node), smaller trees and more interpretable were generated. In the BLTREED model, one subset of *X* can be used to generate the tree and other subsets were used to fit models in terminal nodes (these subsets can be joint and/or disjoint). In the Bayesian approach, *θ*_*i*_ = *B*_*i*_ shows the regression coefficients for the logistic model fitted in an *i*th terminal node.

The recursive stochastic process using a tree-generating stochastic process for tree growing (*p*(*T*)) is as follows [42, 43]:

1. Start from *T* that has only a root node (terminal node *η*)
2. Calculate the probability for splitting node *η* as follows:

(2) $$\begin{array}{c} P_{\text{Split}}=\alpha {\left(1+d_{\eta }\right)}^{-\beta }, \end{array}$$

where *d*_*η*_ is the depth of the node *η*, *α* is the base probability of tree growth of splitting a node, and *β* is the rate that determines the propensity to split decreases with increased tree size.

Actually, *α* and *β* are parameters that control the shape and size of trees, and these parameters provide a penalty to avoid an overfitting model

(3) If the node *η* splits into left and right nodes according to the distribution of  *p*_RULE_(*ρ* | *η*, *T*), then let *T* as the newly created tree from step 3 and reapply steps 2 and 3 to the new children nodes

The BLTREED model was fitted based on standardized data. So, the same prior distribution can be used independently for parameters in the terminal nodes, and they were considered a multivariate normal distribution with zero mean and variance matrix proportional to the identity for these parameters [43, 54].

Posterior distribution function *p* (*T* | *X*, *y*) was computed by combining the marginal likelihood function *p* (*Y* | *X*, *T*) and tree prior *p* (*T*) as follows:

(3) $$\begin{array}{c} P\left(T\;|\;X,y\right)\propto p\left(y\;|\;X,T\right)p\left(T\right). \end{array}$$

In this study, no informative priors were considered. The priors were uniform on variables at a particular node, and all possible splits for variables.

Where *p* (*Y* | *X*, *T*) is as follows:

(4) $$\begin{array}{c} P\left(Y\;|\;X,T\right)=\int p\left(y\;|\;X,\Theta ,Τ\right)p\;\left(\Theta \;|\;T\right)\;d\Theta =\overset{K}{\underset{i=1}{\prod }}\int \overset{n_{i}}{\underset{h=1}{\prod }}p\left(y_{ih}\;|\;x_{ih},B_{i}\right)p\left(B_{i}\right)dB_{i}, \end{array}$$

which *p*(*y* | *X*, Θ, *Τ*), (*y*_*ih*_, *x*_*ih*_), and *n*_*i*_ show the data likelihood function, observed values for *h*th observation in *i*th node, and the number of observations in *i*th node, respectively. The integral of equation four has no closed form, so the Laplace approximation was used to solve it [43, 54].

Chipman et al. [42, 43] utilize a Metropolis-Hastings algorithm to simulate equation (3) for finding trees with the high posterior distribution. The Metropolis-Hastings algorithm simulates a Markov chain sequence of trees, namely, *T*^0^, *T*^1^, *T*^2^, ⋯.

The simulation algorithm was implemented with multiple restarts for reasons mentioned in Chipman et al. [42, 43].

#### 2.5.2. Classification and Regression Trees (CART)

Breiman et al. proposed the CART model [55]. The CART algorithm generates a tree using a binary recursive partitioning, and the tree-generating process contains four steps: (1) tree growing: tree growth is based on a greedy search algorithm, and this algorithm generates a tree by sequentially choosing splitting rules. The CART algorithm uses traditional splitting functions for choosing splitting rules (entropy and Gini index). (2) Tree-growing process continues until none of the nodes can split. (3) Tree pruning: this tree algorithm uses the cost-complexity pruning method for tree pruning to avoid overfitting. This pruning method generates a sequence of pruned trees, and each tree in this sequence is an extension of previous trees. (4) Best tree selection: CART uses an independent test dataset or cross-validation to estimate the prediction error of each tree and then selects the best tree with the lowest estimated prediction error.

### 2.6. Data Analysis

The BLTREED model and classic CART algorithm based on the two splitting functions like entropy and Gini index (after that, we named the CART method-based Gini index as CART1 and CART method-based entropy as CART2) were fitted by using predictor variables such as hemoglobin (Hb), mean cell volume (MCV), mean cell hemoglobin (MCH), and red cell distribution width (RDW) for differential diagnosis of *β*TT from IDA.

The BLTREED model fitted using eight restarts with 6000 iterations per restart and a prior standard deviation of 20 for the logit coefficients [54]. For determining the pair of (*α*, *β*), the BLTREED model was fitted with two choices, 0.5 and 0.95 for the *α* parameter, and four choices for *β* (a range 0.5-2 by step 0.5), then select the pair of (*α*, *β*) that generate the best tree with smallest FNR.

Based on the acceptable method of cross-validation in machine learning studies, for assessing the performance of the three models, the dataset was split randomly in the ratio 2 : 1 into a training and a test dataset, respectively, using a stratified random sample to ensure equal allocation of presences and absences (for a classification tree). The model was then fit to the training dataset, and the set of the best trees was determined. For each tree, the posterior predictive distribution was computed for both the training data and the test dataset; this was implemented for each iteration of the BLTREED algorithms, thus incorporating the uncertainty of the model parameters and the data in the evaluation of models. Finally, the predictive performances were calculated based on the confusion matrix of the posterior predictive distribution for both the training and the test dataset [43, 47, 54, 56, 57].

Differential performance of the Bayesian classification tree and CART was evaluated using criteria such as sensitivity (TPR), specificity (TNR), false-negative rate (FNR) and false-positive rate (FPR), positive predictive value (PPV) and negative predictive value (NPV), positive likelihood ratio (PLR) and negative likelihood ratio (NLR), accuracy, Youden's index, and the area under the curve (AUCROC). AUCROC represents the degree of separate ability showing how much the machine learning model can distinguish between the classes (IDA and *β*TT); actually, it is a global measure of diagnostic accuracy. A perfect classification algorithm has an AUCROC = 1. The interpretation of the AUCROC is described as follows: AUCROC > 0.9: excellent differentiation, AUCROC > 0.8: very good differentiation, AUCROC > 0.7: good differentiation, AUCROC > 0.6: sufficient differentiation, AUCROC > 0.5: bad differentiation, and AUCROC < 0.5: classification method is not useful for discriminating between IDA and *β*TT [58, 59]. Criteria such as Youden's index, accuracy, PLR, NLR (an excellent diagnostic test has NLR < 0.1 and PLR > 10), and AUC take both sensitivity and specificity into consideration, so that can present the performance of the model more accurately than other criteria. In addition, AUC values were compared using DeLong et al. method [60]. A *P* value < 0.05 was considered a statistically significant difference.

### 2.7. Software

Data were analyzed by free software (http://gsbwww.uchicago.edu.fac.robert.mcculloch.research.code.CART.index.html) based on Chipman et al. (2002) that was developed for fitting BLTREED model, R 3.0.3 used for fitting CART algorithm (package rpart), computing performance measures (package ePiR and package pROC), and splitting data to training dataset and test dataset (package caTools).

## 3. Results

A total of 537 patients were diagnosed as *β*TT with an average of age (±SD) 22 ± 16.4 including 299 (56%) women and 238 (44%) men, while 370 patients (mean of age (±SD): 29 ± 14.6) were diagnosed as IDA including 293 (79%) women and 77 (21%) men.  Table 1 shows the median and interquartile range (IQR) of laboratory parameters as predictor variables across the type of hypochromic microcytic anemia (*β*TT and IDA).

The tree structure of CART1, CART2, and BLTREED models is shown in Figures 1–3, respectively. The first split of the three methods of classification trees was based on MCV, which showed that MCV has a higher importance value in differentiation between the *β*TT and the IDA. Another predictor that was used as the second splitting variable in tree structure was HB. According to the presented trees, the BLTREED model produced a smaller tree size and was more interpretable than the CART algorithm (Figures 1 and 2). This model showed values of MCV ≤ 72.6 screening the *β*TT patients. The BLTREED model extracted four homogenous subgroups for differentiating between the *β*TT and the IDA (Figure 3).

The predictive performance of models in differentiation between *β*TT and IDA was calculated based on the confusion matrix (Table 2). The BLTREED model, CART1, and CART2 trees showed the high TPR, TNR, PPV, NPV, Youden's Index, and accuracy in differentiation between *β*TT and IDA (Table 3). However, the BLTREED model had a higher accuracy and Youden's index other than CART1 and CART2.

In addition, all the models have NLR < 0.1 that three classification tree algorithms have good diagnostic accuracy for discriminating the patients.  Table 4 shows the AUCs of the three tree models from ROC analysis that were statistically significant (*P* < 0.001) and revealed that all three classification methods had an excellent diagnose accuracy (AUC > 0.9: excellent differentiation) in differentiation between the *β*TT and the IDA. In addition, Figure 4 displays the receiver operating characteristic curves of the BLTREED model, CART1, and CART2 algorithms for the test dataset, and the comparisons of AUC values between the models. According to the exhibited figure, there was no significant difference between the methods (*P* > 0.05).

## 4. Discussion

In this paper, we used the BLTREED model as the differential diagnostic tool for thalassemia diagnosis. In addition, we compare the predictive performance of the BLTREED model as a Bayesian decision tree with the CART algorithm. It is the first study that uses the BLTREED model in the hematological data.

The Bayesian decision tree was used to solve uncertain problems of conventional tree-based methods [43, 54, 61]. This model was implemented by using Hb, MCV, MCH, and RDW as independent variables.

Our dataset included 537 (59%) patients with *β*TT and 293 (41%) patients with IDA. However, there was not any degree of relative imbalance between the IDA and *β*TT classes. [62, 63].

Based on our result, MCV and Hb were the main predictor parameters in differential diagnostic, and it showed that the patient with *β*TT has lower values of MCV.

In previous studies that used the different conventional decision trees for differential diagnosis *β*TT from IDA, the first split of all algorithms was based on MCV. They also concluded that MCV was a significant predictor variable in the discrimination of IDA and *β*TT [32, 36]. The performance of the BLTREED model that was evaluated using sensitivity, specificity, false-negative and positive rate, and positive and negative predictive value exhibited the high performance of the differential diagnosis of *β*TT from IDA. In addition, positive likelihood ratio, negative likelihood ratio, accuracy, and Youden's index showed that BLTREED has good diagnostic accuracy for discriminating the patients. It was indeed classified as 96% of *β*TT patients. Furthermore, AUC as an overall performance index showed excellent and significant accuracy (99, 98) in training and test data, respectively, in differential diagnostic of *β*TT and IDA. BLTREED has also generated a tree with a smaller size, and it is more interpretable other than the CART algorithms and indicated better diagnostic performance.

Our study has a limitation, which should be considered. The investigated patients have included just IDA and *β*TT cases and excluded concomitant diseases and *α*TT cases. Therefore, considering *α*TT patients in the study would affect the performance of the presented models and changed the interpretation of the result. Particularly when only simple hematologic parameters are used like in the present study, it may be difficult to distinguish *α*TT from *β*TT.

Other studies that used different data mining techniques and decision trees based on the frequentist approach of fitting revealed the high performance and accuracy but lower than our result [32, 34–36, 38]. In many studies which had imbalanced datasets, Oversampling Technique (SMOTE) was applied for handling this problem [34, 64].

The BLTREED model improves the classification performance by solving the uncertainty of previous models [43, 54]. The diagnostic performance of the BLTREED was better than other discrimination methods (classification trees or hematological discrimination indices) in past studies for differentiating *β*TT from IDA. These studies are as follows: Setsirichok et al. used a C4.5 decision tree, naϊve Bayes (NB) classifier, and multilayer perceptron (MLP) for classifying eighteen classes of thalassemia abnormality [38]. Bellinger et al. used classification algorithms like the J48 decision tree, support vector machines (SVM), *k*-nearest neighbors (*k*-NN), MLP, and NB for differentiating between *β*TT, IDA, and cooccurrence of these disorders. In this study, the imbalanced dataset was a cause for the weaker performance [34]. AlAgha et al. compared the diagnostic performance of different classification algorithms such as J48, *k*-NN, artificial neural networks (ANN), and NB for classifying *β*-thalassemia carriers. They showed that SMOTE helped decrease the problem of highly imbalanced class distribution and consequently improved the predictive performance [64]. Jahangiri et al. utilized classification tree algorithms such as CHAID, E-CHAID, CART, QUEST, GUIDE, and CRUISE for differential diagnosis of *β*TT from IDA. They indicated that the CRUISE algorithm has the best diagnostic performance similar to the present study, but this classic algorithm uses the greedy algorithm for tree generating and cannot explore the tree space more than the Bayesian tree approaches. Also, many studies compared the diagnostic performance of hematological discrimination indices, and BLTREED showed better performance in comparison to them [16–19, 23, 25–30, 65–80].

## 5. Conclusion

In the present study, the BLTREED model showed excellent diagnostic accuracy for differentiating *β*TT from IDA. According to the advantages of Bayesian tree-based methods like generating a small and more interpretable tree, and lack of uncertainty of different conventional decision trees, this method can be helpful along with other laboratory parameters for discriminating between these two anemia disorders. Also, understanding tree-based methods are easy and do not need statistical experience. So, it can help physicians in making the right clinical decision.

## Figures and Tables

**Figure 1:** The tree structure of the CART algorithm based on the Gini index (blue terminal node: *β*TT and yellow terminal node: IDA).

**Figure 2:** The tree structure of the CART algorithm based on the entropy index (blue terminal node: *β*TT and yellow terminal node: IDA).

**Figure 3:** Decision tree for the BLTREED model (*α* = 0.95, *β* = 1, Log integrated likelihood = 123.43) (blue terminal node: *β*TT and yellow terminal node: IDA).

**Figure 4:** Receiver operating characteristic curves of BLTREED and CART algorithms in the prediction of IDA and *β*TT groups for test dataset.

**Table 1:** Comparison between hematological parameters of study groups using the Mann–Whitney *U* test (data are presented as median (IQR)).

	*β*TT (*n* = 537)	IDA (*n* = 370)	*P*
MCV (fl)	62 (5.4)	72.2 (9.7)	<0.001
MCH (pg)	19.6 (1.8)	21.9 (4.2)	<0.001
Hb (g/dl)	11 (1.6)	10.5 (2.6)	<0.001
RDW (%)	15.7 (1.7)	15.7 (3.3)	0.94

**Table 2:** Confusion table of the BLTREED model and CART algorithm for training dataset and test dataset.

Dataset	Algorithm	Disease status	TP	FP	FN	TN	(TP+TN)
Training	BLTREED	*β*TT	363	25	13	234	597
		IDA	234	13	25	363	
	CART1	*β*TT	366	46	10	213	579
		IDA	213	10	46	366	
	CART2	*β*TT	358	23	18	236	594
		IDA	236	18	23	358	

Test	BLTREED	*β*TT	155	8	6	103	258
		IDA	103	6	8	155	
	CART1	*β*TT	160	33	1	78	238
		IDA	78	1	33	160	
	CART2	*β*TT	159	12	2	99	258
		IDA	99	2	12	159	

**Table 3:** Sensitivity (TPR), specificity (TNR), false-positive rate (FPR), false-negative rate (FNR), positive predictive value (PPV), negative predictive value (NPV), accuracy, Youden's index, positive likelihood ratio (PLR), negative likelihood ratio (NLR), and diagnostic odds ratio (DOR) of the BLTREED model in prediction of IDA and *β*TT groups and their 95% exact confidence interval for training and test dataset.

	BLTREED		CART1		CART2	
Accuracy measure	Training dataset	Test dataset	Training dataset	Test dataset	Training dataset	Test dataset
TPR	97 (94, 98)	96 (92, 99)	97 (95, 99)	99 (97, 100)	95 (93, 97)	99 (96, 100)
TNR	90 (86,94)	93 (86, 97)	82 (77, 87)	70 (61, 79)	91 (87, 94)	89 (82, 94)
FNR	3 (2, 6)	4 (1, 8)	3 (1, 5)	1 (0, 3)	5 (3, 7)	1 (0, 4)
FPR	10 (6,14)	7 (3, 14)	18 (13, 23)	30 (21, 39)	9 (6, 13)	11 (6, 18)
PPV	94 (91, 96)	95 (91, 98)	89 (85, 92)	83 (77, 88)	94 (91, 96)	93 (88, 96)
NPV	95 (91, 97)	94 (88, 98)	96 (92, 98)	99 (93, 100)	93 (89, 96)	98 (93, 100)
Youden's index	87 (80, 92)	89 (78, 95)	80 (72, 85)	70 (57, 79)	86 (80, 91)	88 (77, 94)
Accuracy	94 (92,96)	95 (91, 97)	91 (89, 93)	87 (83, 91)	93 (91, 95)	95 (91, 97)
PLR	10 (7, 14)	13.36 (7, 26)	5.48 (4, 7)	3.34 (2, 4)	10.72 (7, 16)	9.14 (5, 16)
NLR	0.04 (0.02, 0.07)	0.04 (0.02, 0.09)	0.03 (0.02, 0.06)	0.01 (0, 0.06)	0.05 (0.03, 0.08)	0.01 (0, 0.06)

**Table 4:** The area under ROC curve (AUC) of BLTREED and CART algorithms in the prediction of IDA and *β*TT groups for training and test dataset (SE: standard error of AUC; CI: confidence interval).

	BLTREED		CART1		CART2	
	Training dataset	Test dataset	Training dataset	Test dataset	Training dataset	Test dataset
AUC	0.99	0.98	0.93	0.94	0.97	0.97
SE	0.003	0.009	0.011	0.015	0.006	0.011
95% CI	(0.98, 0.99)	(0.96, 0.99)	(0.90, 0.95)	(0.91, 0.97)	(0.96, 0.99)	(0.95, 1)
*P* value	<0.001	<0.001	<0.001	<0.001	<0.001	<0.001

## Data Availability

The datasets used and/or analyzed during the current study are available from the corresponding author on reasonable request.

## Abbreviations

*β*TT: *β*-Thalassemia trait
IDA: Iron deficiency anemia
MCV: Mean corpuscular volume
MCH: Mean corpuscular hemoglobin
RDW: Red Blood Cell Distribution Width
MCHC: Mean corpuscular hemoglobin concentration
RBC: Red blood cell
BLTREED: Bayesian Logit Treed
TPR: Sensitivity
TNR: Specificity
FNR: False-negative rate
FPR: False-positive rate
NPV: Negative predictive value
PPV: Positive predictive value
PLR: Positive likelihood ratio
NLR: Negative likelihood ratio.
